# Autophagy-independent induction of LC3B through oxidative stress reveals its non-canonical role in anoikis of ovarian cancer cells

**DOI:** 10.1038/s41419-018-0989-8

**Published:** 2018-09-17

**Authors:** Eswara Murali Satyavarapu, Ranjita Das, Chandan Mandal, Asima Mukhopadhyay, Chitra Mandal

**Affiliations:** 1 Cancer Biology and Inflammatory Disorder Division, Council of Scientific and Industrial Research-Indian Institute of Chemical Biology, 4, Raja S.C. Mallick Road, Kolkata, 700032 India; 2 Bose Institute, P 1/12, C. I. T. Road, Scheme – VIIM, Kolkata, 700054 India; 3 Tata Medical Center, 14 MAR, Rajarhat, Kolkata, 700156 India; 4 Northern Institute for Cancer Research, Newcastle University, Newcastle, UK

## Abstract

Cancer cells display abnormal redox metabolism. Autophagy, anoikis and reactive oxygen species (ROS) play a regulatory role during metastasis. LC3 is a well-known essential molecule for autophagy. Therefore, we wanted to explore the molecular interplay between autophagy, anoikis, and ROS in relation to LC3B. We observed enhanced LC3B level along with increased expression of p62 and modulation of other autophagy-related molecules (Atg 3, 5, 7, 12, 16L1 and Beclin1) by inducing oxidative-stress in ovarian cancer cells using a ROS-producing pro-oxidant molecule. Surprisingly, enhanced LC3B was unable to induce autophagosome formation rather promoted anoikis. ROS-induced inhibition of autophagosome-formation is possibly due to the instability of autophagy initiator, ULK1 complex. Moreover, such upregulation of LC3B via ROS enhanced several apoptotic molecules. Silencing LC3B reduced these apoptotic molecules and increased when overexpressed, suggesting its role in apoptosis. Furthermore, LC3B-dependent apoptosis was decreased by inhibiting ROS, indicating a possible link between ROS, LC3B, and apoptosis. Additionally, ROS-induced enhanced LC3B promoted detachment-induced cell death (anoikis). This was further reflected by reduced cell adhesion molecules (integrin-β3 and focal adhesion kinase) and mesenchymal markers (snail and slug). Our in vitro experimental data was further confirmed in primary tumors developed in syngeneic mice, which also showed ROS-mediated LC3B enhancement along with reduced autophagosomes, integrin-β3 and focal adhesion kinase ultimately leading to the decreased tumor mass. Additionally, primary cells from high-grade serous carcinoma patient’s ascites exhibited LC3B enhancement and autophagy inhibition through ROS which provided a clinical relevance of our study. Taken together, this is the first evidence for a non-canonical role of LC3B in promoting anoikis in contrast to autophagy and may, therefore, consider as a potential therapeutic target molecule in ovarian cancer. Taken together, autophagy-inhibition may be an alternative approach to induce apoptosis/anoikis in cancer.

## Introduction

Autophagy is the lysosomal degradation process of cellular components for renewal of energy needed for cell survival during stress conditions^1^. This process is controlled by highly conserved autophagy-related proteins (Atg’s)/p62(sequestosome1)/LC3. Autophagy and epithelial–mesenchymal transition (EMT) play an important role in cancer progression^2^.

Anoikis is a process of detachment-induced programmed cell death in anchorage-dependent cells^3^. EMT is a complex dynamic reversible-process, where cancer cells acquire mesenchymal characteristics, the hallmark of anoikis-resistance, crucial for metastasis^3–5^. Enhanced adhesion molecules are also correlated with anoikis-resistance^6^. Enhanced anoikis-resistance and autophagy are coupled cellular processes crucial for metastasis^7^. Therefore, overcoming anoikis-resistance and inhibiting autophagy would be the ideal therapeutic approach.

However, the molecular-interplay between all major processes related to autophagy and anoikis has not fully deciphered, which might help to discover the specific-target. The LC3 subfamily is considered as the marker-molecule of autophagy^8^. However, the involvement of LC3 in anoikis has not been fully deciphered in cancer. Considering the vital importance of autophagy and anoikis in metastasis, we explored the possible role and molecular mechanism of LC3 in anoikis using ovarian cancer (OC) as a model system. OC is the leading cause of death due to late diagnosis and early metastasis into the abdominal peritoneum/omentum^9^. Therefore, the major task is to search the molecule(s) that could kill a primary tumor and target the metastasized-cells.

Here we provided evidence for a novel non-canonical role of a universal autophagy marker (LC3B) in anoikis. We observed enhanced LC3B and other autophagy-related molecules by inducing oxidative-stress in OC cells using a ROS-producing pro-oxidant molecule. Enhanced-LC3B was unable to induce autophagosome formation possibly due to decreased ULK1-complex. ROS-induced enhanced-LC3B also increased apoptosis. Additionally, LC3B inhibited cell adhesion molecules/mesenchymal-markers, leading to anoikis. Furthermore, in vitro study revealed ROS-dependent enhanced-LC3B reduced the tumor-growth. A similar effect was also observed with primary-cells from patients. Here we demonstrated a unique role of LC3B in vitro/in vivo/ ex vivo in inducing anoikis.

## Results

### A pro-oxidant molecule, mahanine induces ROS in ovarian cancer

We have previously established mahanine as a pro-oxidant molecule in various types of cancers except OC^10^. Therefore, we have used this ROS producing agent to explore the molecular interplay between autophagy, anoikis and ROS. Here we found, mahanine induced four-fold enhanced-ROS within 10 min which gradually decreased with time in PA1 **(**Fig. 1a**)**. ROS was increased in a dose-dependent manner with the highest production at 16.5 µM **(**Fig. 1b**)**. Cells pretreated with a ROS-scavenger, N-acetyl-cysteine (NAC) for 60 min showed reduced ROS **(**Fig. 1c**)**.

**Fig. 1:** Oxidative stress induces LC3B but unable to form autophagosomes. **a** PA1 cells were exposed to a pro-oxidant molecule (mahanine, 16.5 µM) for 0–30 min and stained with H_2_DCF-DA. Mean fluorescence intensity (MFI) emitted by each cell/event was measured by FACS. Mahanine was purified from an Indian medicinal plant as described in Supplementary Fig. S1. **b** PA1 were exposed to different doses of mahanine for 10 min processed similarly. **c** Cells were pre-incubated with NAC (2.5 mM, 60 min) and washed. These cells were exposed to mahanine (16.5 µM) for 10 min and processed. **d** RNA was isolated from treated and untreated cells and RT-PCR was performed using LC3B-specific primers. **e** PA1 and OVCAR3 were treated with different doses of mahanine for 24 h and were analyzed by western blot using anti-LC3B and anti-p62 antibodies. **f** Treated and untreated PA1 cells were allowed to attach on the coverslip and immune-stained with anti-LC3B and anti-p62 antibodies and green color was seen using fluorescence-conjugated secondary antibody. **g** PA1 cells were pre-incubated with NAC for 1 h before treatment with mahanine (24 h). Proteins were isolated and analyzed by western blot using specific antibodies. The data represented as the mean ± SD of three independent experiments.‘*represented the significant difference of *p* < 0.05

### Oxidative-stress enhanced LC3B-II expression but unable to form autophagosomes

In cancer microenvironment, autophagy plays the supporting-role for survival by wrapping the unfolded/inactive-proteins/damaged-organelles into autophagosomes, which fuse with lysosomes and forms autophagolysosomes^1^. Moreover, ROS can regulate the autophagic response^11^. Accordingly, we checked the status of a universal-marker of autophagy (LC3B), as a master-molecule, after inducing oxidative-stress in OC cell. An increased genetic-expression of LC3B was observed in PA1 **(**Fig. 1d**)**. Conversion of LC3B-I to LC3B-II is an essential event for autophagosome-formation to induce autophagy. Accordingly, we monitored the LC3B-II status in anoikis-resistant (PA1) and drug-resistant (OVCAR-3) after ROS-induction. We demonstrated a significant enhancement of LC3B-II (Fig. 1e). Lacking green-punctates suggested inhibition of autophagosome-formation as observed by immunofluorescence **(**Fig. 1f**)**. Our result suggested that ROS-induced LC3B possibly play a different role other than autophagy.

### Oxidative stress enhanced p62, an autophagy substrate, supporting inhibition of autophagy

During stress-conditions, enhanced p62 identifies unfolded/inactive proteins and transfer into autophagosomes by binding with LC3-II^12^ and degrades after autophagolysosome-fusion. Therefore, decreased p62 is an indicator of successful autophagy. However, mahanine-treated PA1/OVCAR-3 exhibited a dose-dependent enhancement of p62 **(**Fig. 1e**)** with reduced punctates **(**Fig. 1f) indicating inhibition of autophagy despite the presence of ROS.

To confirm the enhanced induction of LC3B/p62 is due to ROS, we have pretreated the cells with NAC which showed decreased LC3B-II/p62 levels in mahanine-treated cells, suggesting ROS-dependence **(**Fig. 1g**)**.

### Oxidative stress inhibits autophagy

Oxidative-stress enhanced the LC3B but unable to form the cytoplasmic punctates (autophagosomes, Fig. 1f). Next, we explored the role of ROS in autophagy. Being acidic in nature, autophagolysosomes are detected using acridine-orange^13^. Mahanine-treated PA1/OVCAR-3 exhibited decreased red-fluorescence, suggesting inhibition of autophagy **(**Fig. 2a, b**)**. However, in presence of lysotracker, mahanine-treated cells showed no apparent changes in the intensity of red-fluorescence indicating unaltered lysosomal-acidity **(**Fig. S2a**)**. Late-endosomal and lysosomal membranes-protein (LAMP2) level also remain unchanged indicating no effect of mahanine on lysosomes **(**Fig. S2b**)**.

**Fig. 2:** ROS induces autophagy-related molecules but inhibits the autophagosome formation. **a**, **b** PA1 and OVCAR-3 (5 × 10^5^ cells/well) were treated with different doses of a pro-oxidant agent (mahanine, 24 h) to induce oxidative stress. They were stained with acridine orange as discussed in methods and analyzed by FACS. Acidic vacuoles were measured by decreased relative MFI of red fluorescence where MFI of untreated cells was considered as 100 and compared with treated cells. **c** PA1 cells (5 × 10^5^ per well) were incubated with mahanine, stained with an autophagosome specific green reagent and analyzed by FACS. **d** Mahanine-treated (24 h) OVCAR-3 cells were stained with green reagent and processed similarly. **e** PA1 cells (1 × 10^4^ per well) after attachment on the coated glass coverslip were treated either with mahanine or chloroquine alone or in combination for 24 h, stained similarly and visualized. Green dots representing autophagosomes were captured with fluorescence microscope; scale bar: 100 μm. **f** Number of autophagosomes (green dots) in the above experiment was counted per 100 cells in each case. **g** PA1 cells (5 × 10^5^/well) were treated with either chloroquine alone or with both chloroquine and mahanine combination. These cells were stained with green reagent and analyzed by FACS. **h** Cells were exposed to increasing concentrations of mahanine for 24 h. Total RNA was isolated and RT-PCR was performed using specific primers. **i** Untreated and treated cells (24 h) were sonicated, cell lysates were electrophoresed and analyzed by western blot using specific antibodies. **j** Cell lysate as described above was analyzed by western blot using the anti-Atg12 antibody that can specifically detect Atg5–Atg12 conjugate. **k** Cell lysate as described above was analyzed by western blot using anti-Atg16L1 antibody. **l** Total protein from untreated and mahanine-treated (24 h) PA1 cells was co-immunoprecipitated with anti-Atg5 antibody and immunocomplex was analyzed with anti-Atg16L1and anti-Atg12 antibodies separately. **m** Cells were allowed to attach coverslip and transfected with EGFP-LC3B plasmid and then treated with mahanine and chloroquine separately for 24 h. Images were captured by fluorescence microscope; arrows representing the green punctuate (representing autophagosomes). Zoomed-in insets were provided for a representative cell. **n** Cell lysate as described above was analyzed by western blot using specific antibodies. **o** Total protein from untreated and mahanine-treated (24 h) PA1 cells was co-immunoprecipitated with anti-p-ULK1(ser 757) antibody and immunocomplex was analyzed with anti-Atg13 and anti-FIP200 antibodies. Initiation of autophagy is mediated by the unc-51–like autophagy-activating kinase 1/2 complex (ULK1/2–Atg13–FIP200–Atg101)^19^. These data were derived from three individual experiments and mean ± SD was indicated.‘*represented the significant difference of *p* < 0.05

### Oxidative-stress reduces the number of autophagosomes

Next, we have used specific autophagosomes detecting cationic-amphiphilic tracer dye which emitted green fluorescent^14,15^. FACS-analysis revealed a dose-/time-dependent decrease in green-fluorescence in PA1 in presence of ROS **(**Fig. 2c**)**. A similar dose-dependent decreased in green-fluorescence was found in OVCAR-3, indicating a reduced number of autophagosomes **(**Fig. 2d**)**.

Moreover, microscopic analysis exhibited a decreased number of green-dots in mahanine-treated PA1 reflecting a reduced number of autophagosomes **(**Fig. 2e, f**)**. Additionally, we used serum-starved cells as a positive-control for autophagy^16^. As expected, we observed many green-dots confirming enhanced-autophagy under stress-condition **(**Supplementary Fig. S2c–d**)**.

### No role of oxidative-stress in lysosomal-fusion step

Chloroquine, a known inhibitor of autophagosome-lysosome fusion, leads to enhanced-autophagosomes indicating autophagy inhibition^17^. We already have demonstrated decreased autophagy in mahanine-treated cells **(**Fig. 2c, d**)**. Accordingly, we wanted to check whether mahanine is also an inhibitor of autophagosome-lysosome fusion like chloroquine. Therefore, cells were treated with chloroquine in absence/presence of mahanine. As expected, chloroquine-treated cells showed increased-autophagosomes (Fig. 2e, f). Interestingly, in presence of mahanine, chloroquine was unable to further enhance the autophagosomes. Therefore, mahanine is possibly not inhibiting autophagosome-lysosome fusion like chloroquine **(**Fig. 2g**)**. It may act in a different way to inhibit the autophagy.

### Mahanine alters the expression of other autophagy-related molecules (Atg’s)

By now, we have demonstrated that oxidative-stress reduces the number of autophagosomes even in presence of enhanced-LC3B (Figs. 1 and 2). Therefore, next obvious question was to search the status of other Atg-molecules involved in autophagosome-formation. To our surprise, the enhanced genetic expressions of Atg3/5/7/12 and Beclin1 were observed in mahanine-treated cells (Fig. 2h). A dose-dependent enhancement of Atg7, Atg12, Atg3, Atg5 and Beclin1-proteins were also found (Fig. 2i). However Atg3 level was decreased at the highest dose. Altogether, despite enhancement of all these molecules, mahanine inhibited autophagy.

LC3 and Atg12 are two ubiquitin-like proteins facilitating in ubiquitin-like conjugation systems and play a central role in autophagosome-formation^18^. Though we demonstrated an individual increase of Atg5 and Atg12, there was a reduction in Atg5–Atg12 complex in treated-cells **(**Fig. 2j**)**. Moreover, mahanine-treatment decreased Atg16L1 in PA1 **(**Fig. 2k**)**. Furthermore, the co-immunoprecipitation showed a decreased association of Atg5–Atg12/Atg16L1-conjugate **(**Fig. 2l**)**.

### Overexpression of LC3B unable to induce autophagosomes

Next, we confirmed the inhibition of autophagosome-formation even with overexpressed-LC3B in mahanine-treated cells. Accordingly, EGFP-LC3B plasmid transfected PA1 were treated either with mahanine or chloroquine separately. No green-dots were found in mahanine-treated cells even in LC3B-overexpressed condition, confirming oxidative-stress reduced autophagosomes **(**Fig. 2m**)**. In contrast, many green-dots were observed in chloroquine-treated cells.

### Inhibition of ULK1complex formation by mahanine

ULK1, a mammalian serine/threonine-protein kinase, has an important role in autophagy initiation^19,20^. FIP200 and ATG13, two additional proteins, are necessary for the stability of ULK1 and its localization to the pre-autophagosome. Phosphorylation at Ser757 of ULK1 reduces its affinity towards Atg13.

We demonstrated decreased phosphorylation of ULK1(Ser757) in mahanine-treated cells. Both Atg13/FIP200 were also down-regulated suggesting instability of ULK1-complex **(**Fig. 2n**)**.

Most importantly, co-immunoprecipitation demonstrated the decreased association of FIP200 with p-ULK1(Ser757), suggesting some defect in recruitment of ULK1-complex and subsequent inhibition of autophagosome-initiation **(**Fig. 2o**)**. This might be the possible explanation for why mahanine was unable to form autophagosome.

### Oxidative-stress inhibits proliferation of OC cells

Oxidative-stress leads to increased LC3B and other autophagy-related molecules but ultimately inhibits the autophagy **(**Figs. 1 and 2**)**. Since autophagy is required for survival of cancer cells^11^, we checked the status of oxidative stress in cell death. We found mahanine exhibited significant anti-proliferative activity both in PA1 and OVCAR-3 **(**Fig. 3a); IC_50_ values being 11 and 32 μM, respectively. We routinely observed that adherent treated-cells were detached and float in suspension and became homeless with no cell–cell contacts. Drastic morphological change with the complete collapse of their shape and density was observed **(**Fig. 3b–i**)**.

**Fig. 3:** LC3B mediates enhanced apoptosis through ROS in ovarian cancer cells. **a** PA1 and OVCAR-3 cells were exposed to varying concentrations of a pro-oxidant agent (mahanine, 48 h) to induce oxidative stress. Growth-inhibitions were assessed by MTT assay. Cell viability was calculated as the percentage relative to untreated cells which were considered as 100%. **b** Floating cells in mahanine-treated wells were removed and then phase-contrast images were captured. It shows the collapse of morphology in mahanine-treated cells; scale bar: 100 μm. **c** PA1 and OVCAR-3 were exposed to mahanine and stained with FITC-Annexin-V and PI and analyzed by flow cytometry. **d** Mahanine-treated cells were stained with DAPI. Arrow indicates the condensed or fragmented nucleus (scale bar: 50μm). **e** RT-PCR was performed using specific primers (Caspase3, Capase9, Bax and Bcl2) with total RNA isolated from treated and untreated cells then electrophoresed. **f** Cell lysate as described above was analyzed by western blot using anti-PARP antibody. **g** NAC-pretreated PA1 cells were exposed to mahanine and analyzed by western blot with the anti-PARP antibody. **h** NAC-pretreated PA1 cells were incubated with mahanine and cell death was measured with PI and analyzed by FACS. **i** The reversal of cell death and regain of cell shape and density was also visualized by phase-contrast images after removing floating cells. Arrow represents the live cell colonies in a NAC-pretreated mahanine-treated cell. **j** Cells were transfected with LC3B-siRNA and knocked down of LC3B was confirmed by western blot. **k** LC3B-siRNA transfected and un-transfected cells were exposed to mahanine. RNA was isolated. mRNA levels of apoptotic/anti-apoptotic molecules were analyzed by RT-PCR using specific primers. **l** Proteins were isolated from LC3B-knocked down cells and analyzed by western blot using anti-PARP antibody. **m** PA1 was either transfected with LC3B-siRNA or with EGFP-LC3B and exposed mahanine and stained with Annexin-V-PE and 7-AAD. These were analyzed by flow cytometry. **n** RNA was isolated from mahanine-exposed EGFP-LC3B transfected and un-transfected cells and analyzed by RT-PCR using specific primers to check their gene expression changes. **o** Cell lysate from LC3B-overexpressed cells was analyzed by western blot using anti-PARP antibody. LC3B overexpressed cells showed different PARP cleavage pattern. Both cleaved bands (89 and 55 kDa) were quantified using ‘ImageJ’ software and represented in the bar graph. These data were derived from three individual experiments and mean ± SD was indicated. ‘*’represented the significant difference of *p* < 0.05

### Oxidative stress induces apoptosis

Increased annexin-V positivity from ~ 2 to ~18% in mahanine(24 h)-treated PA1 suggested early apoptosis through loss of membrane integrity **(**Fig. 3c**)**. The number of annexin-V/PI-positive cells was further increased to ~64% indicating late apoptosis. In contrast, a very few cells exhibited only PI-positivity reflecting minimal necrosis. OVCAR-3 exhibited similar apoptosis under similar conditions.

Moreover, DAPI-staining showed fragmented/condensed nucleus suggesting mahanine-induced apoptosis **(**Fig. 3d**)**. Furthermore, the dose-dependent increased caspase-3, caspase-9, Bax, decreased anti-apoptotic molecule (Bcl2) and cleaved PARP at 89 kDa confirmed apoptosis after mahanine-treatment **(**Fig. 3e, f**)**.

Next, we found that NAC significantly rescued mahanine-induced apoptosis as evidenced by reduced PARP cleavage **(**Fig. 3g**)** and decreased PI-positivity **(**Fig. 3h**)**. Moreover, NAC-pre-incubation of mahanine-treated cells restored morphology, shape, and density to almost 80% as exhibited by phase-contrast images suggesting ROS-dependent apoptosis in mahanine-treated cells **(**Fig. 3i**)**.

### LC3B mediates enhanced apoptosis through ROS

Since ROS-induced enhanced-LC3B did not exhibit any role in autophagy, next we investigated its relationship with apoptosis. We observed LC3B-knocked down cells reduced the level of LC3B **(**Fig. 3j**)**, reversed the mRNA levels of caspase-3, caspase-9, Bax, Bcl2 **(**Fig. 3k**)** and PARP cleavage by western blot **(**Fig. 3l**)**. Mahanine-induced higher annexin V/7-AAD^+vity^ (~ 12.5%) is also reduced to ~ 2% when LC3B was silenced indicating the role of LC3B in oxidative stress-induced apoptosis **(**Fig. 3m**)**.

In contrast, overexpression of LC3B enhanced apoptotic cell death from ~12.5 to ~71.2%, which further validated the involvement of LC3B. Moreover, mahanine-treated LC3B overexpressed cells also exhibited further decreased Bcl2 **(**Fig. 3n**)**, increased caspase-3, caspase-9 and Bax **(**Fig. 3n**)**. Additionally, after overexpression of LC3B, we found increased PARP cleavage **(**Fig. 3o**)**. Interestingly, an additional 55 kDa band along with the main 89 kDa cleaved PARP were observed. The pattern of PARP cleavage is possibly due to the different enzymes responsible when more amount of LC3B present^21^. Taken together, we have established a cross-talk between ROS, enhanced-LC3B and apoptosis.

### Mahanine inhibits migration and deregulates EMT markers

Autophagy activation is essential for cancer cell migration/invasion requiring for EMT^22^. Therefore, we checked the status of EMT-related molecules in these stress-induced cells. We found that mahanine significantly inhibited the migration of both PA1 and OVCAR-3 **(**Fig. 4a, b**)**. The mRNA expression of epithelial (E-cadherin) and mesenchymal (snail/slug) markers were decreased in mahanine-treated PA1 **(**Fig. 4c**)**. Reduced E-cadherin, snail and slug proteins were observed **(**Fig. 4d, e**)**.

**Fig. 4:** Mahanine reduced both epithelial and mesenchymal markers in LC3B-dependent manner and induces anoikis. **a** PA1 and OVCR3 cells were seeded in 6-well plate and grown up to > 90% confluent. A confluent monolayer of both cells was scraped with the micropipette tip and exposed to the mahanine. Cells migrated to the wounded region were assessed by phase-contrast microscopy. **b** The inhibition of migration was expressed by calculating the area of a wound as the relative percentage in comparison to untreated cells. **c** Cells were treated with increasing doses of mahanine and RT-PCR (for genetic expression) was performed using specific primers. **d** Protein was isolated from mahanine-treated cells and analyzed by western blot using anti-E-cadherin, anti-slug and anti-snail antibodies separately. **e** PA1 and OVCAR3 cells were treated with mahanine and the expression levels were monitored using fluorescence-tagged antibodies against E-cadherin, snail, and slug by FACS analysis. **f**, **g** Genetic manipulation of LC3B is achieved by transfection of cells with LCB-siRNA or EGFP-LC3B plasmid. These transfected cells were incubated with mahanine for 24 h and RT-PCR was performed with specific primers. Expression levels were compared to un-transfected treated cells. **h**, **i** NAC pre-treated cells incubated with mahanine for 24 h and analyzed by FACS and western blot using specific antibodies. **j** Cells were seeded in TCP or ULA 96 well plate and exposed to mahanine for 48 h. Images were taken with a phase-contrast microscope and sphere formation (PA1) or multi-cellular aggregates (OVCAR-3) were observed. OD < 1.0 representing anoikis-sensitization by mahanine leads to detachment-induced cell death (anoikis). **k** Cell viability was checked by MTT assay. Viability Index (VI) was calculated by taking the ratio of OD in ULA to TCP plates. **l** Mahanine-treated PA1 cells (24 h) were stained with fluorescence-tagged antibodies against integrin-β3 and FAK separately and analyzed by FACS to check the protein levels. **m** LC3B-siRNA transfected cells were incubated with mahanine for 24 h. Integrin-β3 and FAK expression were similarly measured by FACS. **n** LC3 over-expressed cells were treated with mahanine and analyzed by western blot using specific antibodies. **o**, **p**. NAC pre-treated cells were exposed to mahanine (24 h) and the expression levels integrin-β3 and FAK were monitored both by FACS and western blot using specific antibodies. All Individual experiments were repeated for at least three times and mean ± SD was calculated. ‘*’ represented the significant difference of *p* < 0.05

### Oxidative stress-induced LC3B modulates EMT

By now, our results suggested that mahanine-induced LC3B seems to have no role in autophagy but involved in apoptosis. Next, we asked the question, is there any relation between enhanced LC3B and EMT-molecules by LC3B in mahanine-treated cells? Accordingly, LC3B was silenced in PA1 and treated with a ROS-producing agent **(**Fig. 4f**)**. Reduced LC3B increased the genetic expression of snail and slug but there was no significant change in E-cadherin after treatment.

In contrast, LC3B-overexpressed cells in presence of mahanine showed a further decrease of snail and slug compared to mahanine alone indicating LC3B-dependent regulation of mesenchymal markers **(**Fig. 4g**)**. However, E-cadherin level was not changed even after LC3B overexpression suggesting no involvement of LC3B and intermediate EMT phenotype in this context.

Furthermore, in presence of mahanine, NAC-pretreated cells showed a reversal in slug and snail expression suggesting the involvement of ROS in decreasing mesenchymal phenotype by accumulating LC3B (Fig. 4h, i).

All these observations indicate the role of accumulated LC3B in inducing anoikis possibly at the transcriptional level.

### Mahanine induces detachment-induced cells death (anoikis)

Decreased mesenchymal phenotype generally leads to anoikis in cancer cells^3^. We demonstrated that mahanine induces apoptosis **(**Fig. 3**)** and downregulates mesenchymal phenotype **(**Fig. 4c–i**)**. This again raised the possibility of its involvement in anoikis. Therefore, we investigated the role of mahanine in the induction of anoikis through LC3B upregulation.

Accordingly, we performed anoikis assay with PA1 and OVCAR-3 in presence/absence of mahanine. In ultra-low attachment plate, oxidative-stress decreased the number and size of PA1-spheroids with smooth surface indicating inhibition of spheroidogenic property **(**Fig. 4j**)**. In contrast, multi-cellular aggregates were observed in OVCAR-3. However, mahanine-treated cells showed slightly enhanced cell death in ultra-low attachment plate compared to adherent-plate. The viability-index (VI) were 0.89 and 0.78 in treated-PA1 and OVCAR-3 respectively representing anoikis-sensitization indicating the involvement of mahanine in anoikis **(**Fig. 4k**)**.

### Enhanced LC3B sensitizes cells for anoikis

Integrin-β3 and its downstream molecule, focal adhesion kinase (FAK) are decreased during anoikis^23^. We also found decreased integrin-β3 and FAK with accumulated LC3B in mahanine-treated cells (Fig. 4l). When LC3B was silenced, mahanine-treated PA1 showed the enhanced integrin-β3 and FAK indicating increased cell–cell contacts **(**Fig. 4m**)**. Moreover, over-expressing LC3B resulted in an additional decrease of integrin-β3/FAK in mahanine-treated PA1 (Fig. 4n) confirming the involvement of LC3B in detachment of PA1 leading to apoptosis.

Moreover, in NAC pre-treatment, mahanine increased the expression of integrin-β3/FAK (Fig. 4o, p). This reversal suggested that mahanine-induced oxidative stress via accumulation of LC3B possibly take part in the regulation of anoikis-related molecules. Therefore, we could conclude that accumulated-LC3B plays an important role to kill the cancer cells via anoikis demonstrating its non-canonical role.

### Oxidative-stress inhibits tumor growth in syngeneic mice

To confirm the physiological relevance of our experimental data, we generated a syngenic mice model of OC by injecting ID8 cells. Mahanine inhibited the tumor growth (6–8 fold) **(**Fig. 5a, b**)**. There was no decrease in the body weight **(**Fig. 5c**)**. Moreover, the primary cells from treated-tumor mass showed higher PI positivity (~3-fold) signifying accumulation of dead cells **(**Fig. 5d**)**. Furthermore, in corroboration with in vitro findings, these primary cells from treated-mice showed increased ROS (Fig. 5e) and LC3B accumulation **(**Fig. 5h**)** along with reduced autophagosomes number (Fig. 5f) and anoikis-resistance molecules (integrin-β3/FAK, Fig. 5g**)**. This in vitro evidence further strengthened ours in vitro findings.

**Fig. 5:** Mahanine upregulated LC3B, inhibited autophagy and induced anoikis resulting in reduced tumor-growth in the syngenic mouse model. **a** Representative images of mahanine (70 mg/kg/day, 14 days of consecutive treatment) or vehicle (10% ethanol, *i.p*.) treated tumors in BALB/c mice (*n* = 10) generated by injecting ID8 cells (*s.c*; 7 × 10^6^; in 100 µL PBS, matrigel in 1:1) in the left flank; arrows showing tumors attached to the subcutaneous region of mice after dissection. **b** Mean of tumor volume in mm^3^ measured at the end of treatment period (14 days) and compared with untreated. **c** Body weights (grams) of both untreated and treated mice were measured on every alternate day during the treatment period plotted on the graph. **d** Primary cells were isolated from tumors and measured the apoptotic cells by PI staining. ~ 3-fold increase PI positivity found in treated tumor mass compared to untreated). **e** Primary cells stained with H_2_DCF-DA for the measurement of the ROS by FACS and found ~1.5 fold increased ROS. **f**. Primary cells were stained with a green reagent to measure autophagosomes by FACS which shows ~ 50% reduced autophagosomes. **g** Primary tumor cells were incubated with fluorescence-tagged anti-integrin-β3 and anti-FAK antibodies, analyzed by FACS and represented as relative MFI. **h** Tumors tissues from both treated and untreated animals were collected, fixed in 5% formalin solution and processed. Thin sections were incubated with anti-LC3B antibody and followed by Alexa Flour 488 conjugated secondary antibody. Slides were visualized using a fluorescence microscope. All Individual experiments were repeated for at least three times and mean ± SD was calculated. ‘*’ represented the significant difference of *p* < 0.05

### Mahanine induces cytotoxicity, inhibits autophagy but up-regulates LC3B-II in primary cells

To evaluate the clinical relevance, primary cells from ascitic fluids of nine patients of different histology/stages/treatment statuses were evaluated for their sensitivity towards mahanine (Table 1). It exhibited anti-proliferative activity, IC_50_ being 14–35 µM (Fig. 6a). Primary cells exhibited complete collapse of their shape/density (Fig. 6b), reduced autophagosome-formation (Fig. 6c) and increased LC3B-II (Fig. 6d) in presence of oxidative stress. This clinical evidence clearly indicates that the ROS-producing agent could be a better therapeutic molecule for treating OC patients.

**Table 1:** Patient related information and IC_50_ values in the primary cells

ID	Age	Stage and histology	Treatment status		Source for primary culture		IHC	IHC	IC_50_ (µM)
			Post op 6 cycles chemo (C + P)	Progression at 6 months	Ascites	Chemo naive	PAX8	WT1	
PCAST-1	65	IIIC HGCS	√	no	√	√	√	√	34.7 ± 0.02
PCAST-3	45	IVC HGSC	√	yes	√	√	√	√	19.6 ± 0.5
PCAST-4	52	IIIC HGSC	√	no	√	√	√	√	28.5 ± 0.08
PCAST-6	52	IIIB (Clear cell)	√	no	√	√	√		23.2 ± 0.02
PCAST-12	40	IIIC (HGSC)	√	no	√	√	√	√	23.2 ± 0.01
PCAST-14	46	IIIC (HGSC)	x	yes	√	√	√	√	22.3 ± 0.02
PCAST-15	56	IIIC (HGSC)	√	no	√	√	√	√	30 ± 0.5
PCAST-16	56	IVB (HGSC)	√	no	√	√	√	√	27.4 ± 0.15
PCAST-17	64	IIIC (HGSC)	x	no	√	√	√	√	14.5 ± 0.15

Clinical data of patient sample/primary cells includes patient age, stage/histology treatment status and origin. We confirmed the epithelial ovarian cancer cells (EOC) by IHC of various markers (PAX8, WT1). PCAST- primary culture ascites; HGSC- high-grade serous cancer; C + P- carboplatin + paclitaxel.

*PCAST* primary culture ascites, *HGSC* high-grade serous cancer, *C+P* carboplatin + paclitaxel

**Fig. 6:** Mahanine up-regulating LC3B through oxidative stress and inhibits cell growth and autophagy in primary cells isolated from patients with high-grade serous histology. **a** Primary cancer cells were isolated from ascitic fluid of nine patients . Cells (1 × 10^4^ /well) were plated, treated with mahanine and processed as described in Fig. 3a. **b** Primary cells from three representative patients (5 × 10^5^ per well in 6-well plates) were treated with mahanine (near to IC_50_ dose). Phase-contrast images showing the collapse of morphology in treated cells (scale bar: 100 μm). **c** Primary cells from three representative patients (PCAST-4, PCAST-14, and PCAST-17) were treated similarly for 24 h and processed to determine the percent autophagosome by FACS, which exhibited reduced autophagosome-formation up to ~ 70%. **d** Primary cells (1 × 10^6^/well) from these patients were treated with mahanine for 24 h. Cell lysates were electrophoresed and analyzed by western blot using anti-LC3B antibodies. **e** Model illustrating the possible mechanism of oxidative stress-induced enhanced LC3B leading to anoikis but inhibited autophagy. A pro-oxidant agent (mahanine) enhanced LC3B via oxidative stress, which induces cell detachment by modulating EMT markers and downregulating cell adhesion molecules like integrin-β3 and focal adhesion kinase (FAK), leading to form homeless cells. Enhance LC3B also induces the apoptotic molecules (caspase-3, caspase-9, Bax and PARP cleavage) and downregulate anti-apoptotic molecule (Bcl2), which induces detachment-induced cell death (Anoikis). Such oxidative stress induces autophagy-related molecules like Atg 3, 5, 7, 12, p62, Beclin1 and LC3B-II, and also inhibits the formation of ULK1 complex, which leads to inhibition of autophagy

## Discussion

The main achievement of our study is to demonstrate a non-canonical role of LC3B in detachment-induced cell death (anoikis) instead of canonical involvement in autophagy, induced by ROS in OC. Mahanine-induced accumulated LC3B sensitized these cells for anoikis by modulating mesenchymal markers and adhesion molecules. These were further supported by in vitro evidence, in which primary cells from treated-mice showed increased ROS, LC3B and reduced autophagosomes, integrin-β3/FAK indicating enhanced anoikis. Additionally, primary cells from patients showed reduced cell growth, enhanced LC3B and inhibition of autophagosome. Taken together, we provide an autophagy-independent novel role of LC3B in mediating anoikis, suggesting as a specific regulatory target.

Abundant availability, structural diversity and non-toxic nature of herbal molecules make them potential source as chemotherapeutics^24^. Mahanine from an edible Indian medicinal plant exhibited apoptosis via ROS in cancers cells with minimal toxicity to normal cells/tissues. It activated death receptor-induced apoptosis in leukaemia, acts as a mTORC1/2 inhibitor in glioblastoma multiform, Hsp90 inhibitor in pancreatic, enhanced tumor suppressor proteins (PTEN/p53) in colon cancers. Moreover, it showed a synergistic effect with clinically-approved drugs and exhibited immunomodulation^25–32^. Encouraged by these observations, we utilized this pro-oxidant molecule to induce oxidative-stress in OC to understand the interplay between autophagy and anoikis. Here, we demonstrated its apoptotic effect even in anoikis-resistant cells and primary cells from syngenic mouse and patients. Therefore, this multi-targeted mahanine may be considered as a promising therapeutic candidate to fight against OC.

Both autophagy and apoptosis are two independent processes, which may or may not influence each other^1^. Caffeine-induced autophagy leads to apoptosis in cancer^33^. In contrast, apoptosis of cancer cells has been demonstrated through autophagy inhibition. Apigenin and sorafenib inhibited autophagy and enhances apoptosis in breast cancer^34^ and hepatocellular carcinoma^35^, respectively. Autophagy-inhibition increases radio-sensitivity in breast cancer^36^. Therefore, autophagy-inhibition may be an alternative therapeutic approach for inducing apoptosis.

Autophagy, a self-eating process, involves the formation of autophagosomes, fusion with lysosomes (autophagosome-lysosome fusion step) and degradation. We have observed that oxidative stress-induced cells exhibited a decreased acid-vacuoles, autophagosomes-specific staining and cytoplasmic puncta indicating inhibition of autophagosome formation. However, mahanine is not involved in autophagosome-lysosome fusion. Therefore, mahanine-induced oxidative stress might reduce autophagy by inhibiting autophagosome formation only.

Out of seven orthologues of LC3/GABARAP family, LC3B is a widely accepted marker for autophagy^37^. Despite inhibition of autophagosome formation, we demonstrated oxidative-stress-induced LC3B accumulation. Moreover, autophagy is usually monitored by Atg’s/Beclin1^38,39^. All these markers were enhanced in presence of ROS, suggesting autophagy. However, we observed inhibition of autophagosome formation even after LC3B overexpression. Thus, oxidative-stress-induced enhanced Atg’s/Beclin1 were not sufficient to induce autophagosome formation as corroborated with others^40^. Again, an increased p62 in mahanine-treated cells possibly suggested autophagy-inhibition.

Initiation of autophagy is mediated by ULK1/2–Atg13–FIP200–Atg101 complex^19^. While investigating the main reason behind oxidative stress-induced inhibition of autophagosome formation; we observed the decreased association of FIP200 with ULK1-Atg13-FIP200 complex, a facilitator of autophagosome biogenesis. Therefore, mahanine-induced oxidative-stress was unable to recruit the initiation-complex which possibly leads to inhibition of autophagosome formation.

During canonical and non-canonical autophagy, the Atg5–Atg12–Atg16L1 complex is essential for LC3-lipidation^41–43^. Although we found increased Atg5/Atg12 in mahanine-treated cells, there was a reduced Atg5–Atg12 complex. Additionally, we also observed dissociation of Atg5–Atg12/Atg16L1 complex, despite enhanced LC3B, which needs further investigation.

Although, LC3B is a marker of autophagy, there are some context-specific contrasting reports^44^. LC3B/LC3 subfamily is not required for autophagosome formation during starvation-induced autophagy but plays some role in autophagosome size/autophagosome-lysosomefusion^45^. Here, we have demonstrated enhanced LC3B-accumulation and inhibition of autophagosome formation in mahanine-treated cells. Therefore, we are proposing an autophagy-independent non-canonical role of LC3B.

Migration and invasion are needed for EMT, during which autophagy is activated^46,47^. Cancer cells expressing more mesenchymal markers show anoikis-resistance and become aggressive^3^. We have observed inhibition of migration and decreased epithelial/mesenchymal markers in mahanine-treated cells where LC3B is accumulated. Silencing LC3B increased mesenchymal marker, whereas overexpression decreased their levels, suggesting the role of accumulated-LC3B in inducing anoikis-sensitization possibly at the transcriptional level. Furthermore, reversal of mahanine-effect on snail/slug expression in NAC-pretreated condition suggested ROS involvement in decreasing the mesenchymal phenotype of these cells.

Cells form spheroids for survival by increasing cell–cell contacts after detachment and become more anoikis resistant^3^. We found this pro-oxidant molecule able to kill OC cells both in attached and suspension conditions. Indeed in suspension, it showed more effect indicating its anoikis-sensitization. Mahanine decreased the spheroid size in PA1 indicating its ability to kill more aggressive cells, giving a hope that it could act as a promising agent even in metastatic/late stages.

Anoikis is integrin-mediated cell death^23^. We found mahanine-induced accumulated LC3B inhibits integrin-β3/FAK confirming its role in anoikis-sensitization. Thus, we demonstrated an important role of LC3B in anoikis with no apparent role in autophagy. Furthermore, silencing LC3B increased the mesenchymal markers without complete loss of epithelial markers in mahanine-treated cells representing intermediate-mesenchymal phenotype, which is more anoikis-resistant and aggressive type^3^. Additionally, mahanine unable to inhibit, indeed, increased the integrin-β3/FAK in LC3B-knocked down and decreased after overexpression, validated the involvement of LC3B in detachment leading to apoptosis. Additionally, reversal of anoikis-resistance molecules in NAC pre-treated cells suggested the probable involvement of mahanine-induced ROS. Therefore, oxidative stress-induced accumulated LC3B plays an important role in inducing anoikis again suggesting its non-canonical role.

Additionally, we demonstrated it’s potent ability to kill primary cells from patients. Although primarily rich in epithelial components, these cultures also have some stromal cells reflecting the true microenvironment, and therefore allow us to study the overall effect of oxidative-stress on both epithelial cells and stromal components. Most of the primary cultures with variable response to ROS were from patients who have not relapsed yet after 6 months of completion of platinum-based chemotherapy after surgery. Interestingly, PCAST-3 and PCAST-14 from patients who were platinum resistant/refractory and recurred/died within 6 months start of treatment, also showed a reasonably good response to ROS. Both patients had tumor characteristics (fibrotic/nodal) during surgery that would indicate a mesenchymal phenotype and cytoreduction could not be achieved. We also generated a few primary cultures from omental tissue (PCT MOM 3–6) obtained from patients of various other histology which generally do not respond well to platinum-based chemotherapy (clear cell, mixed endometrioid, low grade serous and mixed Mullerian tumor) and found ex vivo cytotoxicity to mahanine (IC_50_ 20–30 µM; data not shown). In another ongoing study, we are continuing to explore the effect of mahanine in epithelial/stromal components of solid tumors and to strengthen the correlation between IC_50_ values and LC3B/autophagosomal levels in a larger prospective cohort with matched clinical data.

In conclusion, despite induction of autophagy-related molecules including Atg’s, LC3B and p62, oxidative-stress inhibited autophagy which indicates conventional markers are not universally adequate for autophagy and also suggesting that all these molecules might have some other roles independent of this self-eating process. Moreover, enhanced-LC3B helped in detachment of cells by changing mesenchymal and adhesion molecules which induced anoikis and ultimately cell death even in anoikis-resistance cells (in vitro), primary cells from patients (ex vivo) and reduced tumor growth in vitro.

Taken together, our study was the first to describe circumstances in which LC3B signaling leads to anoikis cell death which could be helpful to manage metastasis. Additionally, these findings highlighted the double-edged role of a pro-oxidant agent which inhibited autophagy and induced apoptosis ultimately giving a hope that it can be potentially helpful for management of OC patient even in the advanced stage.

## Material and methods

### Reagents

All the primary antibodies integrin-β3 (13166), FAK (3285), rabbit IgG, HRP-linked Antibody (7074), β-actin (4970), Autophagy antibody sampler kit (4445), Epithelial–mesenchymal transition (EMT) Antibody Sampler Kit (9782), anti-LC3B antibody (Sigma, L7543) and LC3B-siRNA II (6213) were from Cell Signalling Technology. E-cadherin-FITC (612130), FITC-annexin V (556547), BD cytofix/Cytoperm (554722) and BD Perm/Wash (554723) and ultra-low attachment 96 well plates were purchased from BD Bioscience. Antibody-labeling kit (135–1002), ChemiDoc MP imaging system was from BIO-RAD. Cell culture medium RPMI-1640, MEM, fetal bovine serum (FBS), antibiotic-antimycotic, and trypsin–EDTA were from Invitrogen. 3-(4, 5-dimethylthiazol- 2-yl)−2, 5-diphenyl tetrazolium bromide (MTT), anti-LC3B antibody (L7543), propidium iodide (PI), molecular grade BSA, Tween-20 and dimethyl sulphoxide (DMSO), acridine orange, collagenase, matrigel were from Sigma-Aldrich, USA. Autophagy detection kit (139484) was obtained from Abcam. The EGFP-LC3B plasmid obtained from addgene (11546). BCA protein assay kit, West pico-ECL system was from Thermo Scientific, USA. PVDF membrane was from MILLIPORE, Bedford, MA, USA (Immobilon-P PVDF Membrane# IPVH00010). H_2_DCFDA was purchased from Molecular Probes. Lipofectamine LTX and Plus reagent obtained from Invitrogen USA. Solvents (AR grade, Merk chemicals), HPLC column: RP-C18, 5 µm, 250 × 4.6 mm from Waters.

### Cell cultures

Human OC cell line OVCAR-3 was purchased from ATCC at co-authors lab. PA1 from ATCC was authenticated by STR profiling performed at Lifecode Technologies Pvt. Ltd. (service code: LC-M-321; Nov’2016) and crosschecked with ATCC data bank **(**Supplementary Table 1**)**. They were grown in MEM and RPMI-1640, respectively supplemented with 10% fetal bovine serum (FBS), glutamine (2.2 g/L) and 1% antibiotic-antimycotic (complete medium) at 37 °C with 5% CO_2_.

### Purification and characterization of mahanine

Mahanine was purified from leaves of an Indian medicinal plant, *Murraya koenigii* according to our standard protocol with little modifications^10^ (Fig. 1S). This molecule has been used as a pro-oxidant molecule throughout our study to induce oxidative stress in cancer cells.

### Intracellular ROS measurement

PA1 was treated with mahanine (16.5 µM; 5 × 10^5^/well) for 0–30 min and incubated with H_2_DCF-DA (50 µM) for 30 min at 37 °C in dark. Cells were washed and suspended in PBS. Intracellular ROS was determined by FACS^25^. Similarly, cells were exposed to different doses of mahanine (0–16.5 µM) for 10 min and processed. Furthermore, cells were pretreated with NAC (2.5 mM) for 60 min, washed, treated with the highest dose of mahanine (16.5 µM) for 10 min and processed similarly.

### Reverse transcription (RT)-PCR

Total RNA was extracted from mahanine-treated (0–16.5 µM; 1 × 10^6^ per well; 24 h) cells using RNeasymini kit and reverse transcribed into cDNA with random primers using the Im-Pro-II-Reverse transcription system. PCR assays were carried out with specific forward and reverse primers **(**Table 2**)** using a PTC-100 system^48^. The PCR products were electrophoresed on an agarose gel (1%), stained with ethidium bromide and visualized and pictures were captured with BIO-RAD trans-UV system. Mahanine exposed NAC-pretreated or LC3B-siRNA transfected cells were similarly processed.

**Table 2:** List of primers used in RT-PCR

Target Gene	sequence (5′ to 3′)	Annealing temperature (°C)	product size (bp)
Bax	GGGGACGAACTGGACAGTAA	50	490
	CCTCCCAGAAAAATGCCATA		
Bcl2	GGATGCCTTTGTGGAACTGT	50	479
	GGTGCTTGGCAATTAGTGGT		
Caspase 3	TGGAATTGATGCGTGATGTT	84	460
	TCAAGCTTGTCGGCATACTG		
Caspase 9	GCTTAGGGTCGCTAATGCTG	25	490
	GTGCTGAACATCCCACAATG		
GAPDH	GTCAGGTCCACCACTGACAC	55	225
	GGAAGGACTCATGACCACAG		
LC3B	GGTGAGAAGCAGCTTCCTGT	50	235
	TCTCCTGGGAGGCATAGACC		
Beclin1	GGACACTCAGCTCAACGTCA	45	208
	AGCCTGGACCTTCTCGAGAT		
Atg3	GAGCAACGGCAGCCTTTAAC	25	192
	TCCAAGTTCTCCCCCTCCTT		
Atg5	ACAGATGACAAAGATGTGCT	50	228
	TGGTGTGCCTTCATATTCAA		
Atg7	TGCTATCCTGCCCTCTGTCT	52	193
	GCAAGGAAACCAGCACCATG		
Atg12	AAGTGGGCAGTAGAGCGAAC	52	203
	CACGCCTGAGACTTGCAGTA		
E-Cadherin	TCATGAGTGTCCCCCGGTAT	50	240
	TCTTGAAGCGATTGCCCCAT		
Snail	GAGGACAGTGGGAAAGGCTC	52	248
	TGGCTTCGGATGTGCATCTT		
Slug	CATCTTTGGGGCGAGTGAGT	52	191
	GGCCAGCCCAGAAAAAGTTG		

### Western blot

Mahanine-treated cells (1 × 10^6^ in duplicate, 24 h) were sonicated and centrifuged (10,000 × *g*, 5 min). The supernatants were used as cell lysates^49^. The proteins were quantified with the Thermo scientific BCA protein assay kit. Equal amounts of proteins (40–70 µg) were separated by SDS-PAGE (5–12%) and electrotransferred to nitrocellulose membrane. The membrane was blocked with Tris buffer saline-bovine serum albumin (TBS-BSA; 2–5%) for 5–30 min at 25 °C and probed with the primary antibody. Blots were washed with TBS-Tween-20 followed by incubation with HRP-conjugated secondary antibodies and detected by West-pico ECL system and images was captured by ChemiDoc MP imaging system, with image lab software. Such analysis was similarly performed using NAC-pretreated or LC3B-siRNA/EGFP-LC3B plasmid transfected PA1 and primary cells treated with mahanine. β-actin was used as a loading control.

### Co-immunoprecipitation (co-IP)

Both mahanine treated and untreated cells were sonicated (Qsonica-LLC, XL-2000 series, Newtown, CT, USA)^28^. The cell lysate was centrifuged at 10,000 rpm, 5 min at 4 °C to remove cell debris. Total protein (300 μg/200 μl) was incubated with anti-pULK1(ser757) antibody (1:100) overnight at 4 °C. Immuno-complex was incubated with protein A-sepharose 4B for 3 h at 4 °C and washed with ice-cold phosphate-buffered saline for 3–4 times. The immune complex was resolved by SDS-PAGE (10 %) and identified by appropriate antibodies to check the association with FIP200 and Atg13. Co-IP experiment was repeated using anti-Atg5 antibody (1:100) and processed similarly to check the association with Atg12 and 16L1 using specific antibodies.

### Immunocytochemical staining

PA1 (1 × 10^4^) adhered on poly L-lysine coated coverslip for 3 h and incubated with mahanine (11 µM) and chloroquine (20 µM) for 24 h at 37 °C. Subsequently, they were washed with PBS-0.1% Tween 20 (PBST) and fixed with PFA. Fixed cells were then incubated with goat serum for 1 h at 25 °C and allowed to bind with primary antibodies for overnight at 4 °C. They were visualized by incubation with Alexa Flour 488 conjugated secondary antibodies for 1 h at 25 °C^50^. Images were observed after extensive washing with PBS-T using fluorescence microscope.

### Measurement of acid vacuoles by acridine orange staining

Mahanine-treated cells (1 × 10^6^; 24 h) were stained with acridine orange for 30 min at 37 °C, washed and analyzed by FACS with a 488 nm (blue light) argon laser beam. The red (650 nm) fluorescence was measured.

### Quantification of autophagosomes

This was performed using autophagy detection kit^14,15^. Briefly, PA1 (1 × 10^6^) were treated with mahanine for 12 h/24 h or with autophagy positive control (chloroquine) or both for 24 h. Untreated/treated cells were collected, washed and re-suspended in PBS-5% FBS. Then the green detection reagent was added and incubated at 37 °C for 30 min. Cells were washed and analyzed by FACS. Additionally, OVCAR-3, primary cells from a mouse tumor and three representative patients were processed similarly.

PA1 (5 × 10^5^) were treated with mahanine alone or in combination with chloroquine and similarly stained with a green detection reagent. Images were captured with a fluorescence microscope. The total numbers of green dots per field were counted in five different images per sample from treated/untreated groups. The number of auotphagosomes/100 cells was calculated. In parallel, cells were serum starved for 24 h and processed similarly which served as positive control.

### Transient transfection

Transfection was performed using Lipofectamine LTX and Plus reagent^51^. Briefly, cells (5 × 10^5^) were plated in Opti-MEM (800 μl) for 24 h in a 6-well plate. Plus reagent and LC3B-siRNA or EGFP-LC3B plasmid DNA (1.5 μg) were taken in Opti-MEM (100 μL) in 1:1 ratio and kept at 25 °C for 15 min. LTX (4 μL) in Opti-MEM (100 μL) was added and incubated further for 30 min. This mixture (200 μL) was added to each well and incubated for 6 h. Cells were cultured with the fresh complete medium for another 24 h. Cells were similarly prepared without siRNA/plasmid DNA serving as a control.

EGFP-LC3Band siRNA-transfected cells were incubated with mahanine. RNA and protein were isolated for RT-PCR and western blot analysis respectively. EGFP-LC3B transfected cells were incubated separately with mahanine/chloroquine for 24 h. Images were taken with a fluorescence microscope.

### Cell viability assay

Mahanine-induced cell death was determined by MTT assay^27^. In brief, both PA1 and OVCAR-3 (8 × 10^3^–1 × 10^4^/250 µl per well) were incubated with mahanine (0–50 µM) for 24, 48 and 72 h at 37 °C separately. The medium was discarded and MTT (dissolved in IMDM,100 µg/well) was added (3 h, 37 °C). Formazan crystals formed were dissolved in DMSO and quantified at 550 nm in an ELISA reader and percent of cell viability was calculated. Primary cells from ascites of patients (Table 1) were processed similarly. Both OVCAR-3 (5 × 10^5^ per well in 6-well plate) and primary cells were treated near to IC50 value for 48 h. They were visualized under phase-contrast microscope.

### Annexin V/PI positivity

LC3B-Si-RNA or EGFP-LC3B transfected and untransfected PA1 cells (5 × 10^5^ per well) were incubated with mahanine (0, 11 and/or 16.5 µM) for 24 h at 37 °C^30^. Mahanine-induced apoptosis was determined by suspending these cells in annexin V binding buffer and incubated for 45 min in dark at 25 °C. Annexin-V-FITC/PI (5 µg/mL) or Annexin V-PE/7-AAD (5 µg/mL) were added and kept for 20 min in dark at 4 °C. The acquisition was done in FACS and analyzed by CellQuestPro software. OVCAR-3 cells were also treated with mahanine (0–36 µM) and processed similarly. Additionally, primary cells from a mouse tumor were similarly stained with PI and analyzed. Likewise, PA1 were pretreated for 60 min with glutathione precursor, N-acetyl cysteine (NAC, 2.5 mM) and subsequently exposed to mahanine (0–16.5 µM), stained with PI and analyzed.

### Nuclear staining with DAPI

PA1 (1 × 10^6^) were treated with mahanine (0–16.5 µM, 24 h) and fixed with 4% paraformaldehyde (PFA). They were washed, stained with 4, 6-diamidine-2-phenylindolehydrochloride (DAPI, 1 mg/ml) in PBS for 5 min at 25 °C, washed with PBS and visualized using Leica 6000B microscope. Mahanine (0–36 µM)-treated OVCAR-3 were processed similarly.

### Scratch-wound assay

Both PA1 and OVCAR-3 (1 × 10^6^/ml per well) were cultured to > 90% confluence and scratch-wounds were made by a 10 µL micropipette tip, washed thrice to remove cell debris, and subsequently cultured with mahanine for 24 h. Wound size was calculated and expressed in relative percent compared to untreated cells.

### Fluorescence tagging of antibodies for FACS analysis

Antibodies against Snail/Slug/integrin-β3/FAK were labeled using an antibody labeling kit. Reaction buffer (5 µL), antibody solution (1 mg/ml, 50 µL) and labeling dye (55 µL) were incubated for 60 min at 25 °C. Quencher buffer was added and incubated further for 10 min in dark. These labeled antibodies were used for staining mahanine-treated cells for FACS analysis.

### Anoikis assay

Equal numbers of cells (1 × 10^4^) were seeded both on normal tissue culture plate (TCP) and ultralow-attachment (ULA) 96 well plates separately. They were exposed to mahanine for 48 h and MTT assay was done. The viability index (VI) was calculated which is the ratio of percentage of live mahanine-treated cells in ULA to TCP plates. The VI less than 1.0 represents anoikis sensitization^3^. Untreated cells served as control. Additionally, phase-contrast images were captured for comparison between TCP and ULA plate.

### Syngenic mice model

Female BALB/c mice (*n* = 10, 4–6 weeks old) were injected subcutaneously with mouse ovarian cancer (ID8, 7 × 10^6^) cells. Tumors (~150–200 mm^3^) were generated within seven days. Mice were injected (*i.p*) either with mahanine (70 mg/kg b.wt/day) or vehicle. The tumor size was monitored with screw gauge . Reduction in tumor mass was observed after seven days. However, treatment was continued for another seven days. Tumor tissues were collected after 14 days, dissected and treated with collagenase solution (1 mg/ml)^52^. Subsequently, it was incubated for 2 h at 37 °C in IMDM, centrifuged, washed and re-suspended in the medium. Fibroblasts were removed by 1 h pre-incubation and epithelial cells were used instantly for subsequent experiments.

### Immunohistochemistry

The formalin-fixed mouse tumors were sectioned and processed as previously described^51^. Tissue sections were blocked with 5% BSA in TBST (0.1% Tween 20 in Tris buffer saline) for 30 min and incubated overnight with an anti-LC3B antibody. These slides were washed and incubated with Alexa Flour 488 for 2 h in dark. Finally, they were stained with DAPI and images were captured by fluorescence microscopy.

### Primary cell from ascites

We have developed adherent primary cell cultures from ascitic fluids of nine patients and named as PCAST-1, 3, 4, 6, 12, 14, 15, 16 and 17 (Table 1). Ascitic fluid was collected in the operating room under sterile conditions in patients undergoing primary cytoreductive surgery. Immunocytochemistry/immunohistochemistry was performed in cell blocks from ascetic fluid and formalin-fixed, paraffin-embedded tissues; WT1 and PAX8 staining were performed to confirm Mullerian and epithelial origin histological subtypes of ovarian cancer. Intra-operative tumor distribution and character (peritoneal/fibrosis/nodal) were recorded. In PCAST-3 and PCAST-14 patients (surgery could not be completed due to atypical fibrotic and nodal disease (open and close/palliative surgery). All patients (except PCAST-14 and 17) received 6 cycles of platinum/taxol-based chemotherapy and are undergoing follow up for recurrence and platinum-free interval except for PCAST-14, who died due to progressive disease^52^.

### Ethics approval

All procedures were approved by the animal ethics committee of CSIR-IICB. All samples from patients were obtained with their informed consent for bio-banking. Use of primary tissue material was prior approved by ethics committee of Tata Medical Center review board (Ref. No.: EC/TMC/87/17).

### Statistical analysis

The data shown were representative of three sets of independent experiments. Each experiment was performed in triplicate and the results were analyzed using graph pad Prism (version 5.1). The results were represented as mean ± SD from independent experiments and a significant difference was indicated (‘*’*p* < 0.05).

## Electronic supplementary material

Supplementary table-1: Human cell lines information and supplementary figure legends

Figure S1 Chemical structure of a pro-oxidant agent (Mahanine)

Figure S2

Figure S3
